The article "Epiploic Appendagitis in an Incarcerated Inguinal Hernia: A Case Report and Literature Review" was published in 2022. Journal: Cureus.

# Epiploic Appendagitis in an Incarcerated Inguinal Hernia: A Case Report and Literature Review

**DOI:** 10.7759/cureus.21139

**Published:** 2022-01-11

**Authors:** Najam Husain, Vilomi Bhatia, Muhammed Rahman

**Affiliations:** 1 Colorectal Surgery, University Hospitals of Derby and Burton, Burton upon Trent, GBR; 2 General Surgery, Queens Hospital Burton, Burton upon Trent, GBR

**Keywords:** incarcerated right inguinal hernia, incarcerated appendagitis epiploica, tinea coli, sigmoid colon, appendagitis epiploica, right inguinal hernia

## Abstract

Epiploic appendagitis (EA) is a rare and frequently overlooked cause of abdominal pain. EA within the sigmoid colon in a right-sided inguinal hernia is a rare entity with only a few cases reported. In this article, we present a case of an 80-year-old male with a palpable mass within an incarcerated right inguinal hernia. The patient underwent urgent surgical intervention due to incarceration and the operative findings were of a large indirect inguinoscrotal hernia containing sigmoid colon, with an inflamed epiploic appendage. The colon was reduced into the abdominal cavity and standard tension-free Lichtenstein repair was performed. EA should be a consideration in patients with an acute abdomen as well as those with a painful groin lump. CT is diagnostic; however, emergency surgery should not be delayed for a scan if the hernia is irreducible and tender.

## Introduction

Epiploic appendages may be involved in a number of disease processes such as epiploic appendagitis (EA) due to torsion or venous occlusion or acute and chronic inflammation secondary to diverticulitis. EA is a rare and uncommon cause of abdominal pain, when found in the inguinal hernia sac, the epiploic appendages may appear normal, hypertrophied, inflamed with diverticulitis, or strangulated with necrosis [1]. Its primary presentation results from torsion of the appendage leading to thrombosis of draining vein. This manifests as localised oedema, inflammation and ischemic necrosis, however, it can secondarily be inflamed due to diverticulitis or even a pelvic pathology.

It often presents as non-specific lower abdominal pain, with a predilection in obese middle-aged men, this condition can easily be mistaken for more serious surgical causes of an acute abdomen such as diverticulitis or appendicitis [2]. Finding EA in a hernia sac is extremely uncommon.

This paper aims to outline such a case of EA of the sigmoid colon in an incarcerated right-sided inguinal hernia. To the authors’ knowledge, there are only a few prior cases noted in the literature. Most of the cases are related to the sigmoid colon and a left inguinal hernia.

## Case presentation

We present the case of an 80-year-old man with a known reducible inguinal hernia. He presented to the emergency department complaining of irreducibility for a fortnight. Although he appeared systemically well, he complained of increasing tenderness on the irreducible lump in the right groin. He didn’t have any associated symptoms of bowel obstruction or strangulation. The patient had a past history of hypertension. On physical examination, a large complete right-sided incarcerated inguinal hernia was noted along with a palpable hard mass within the hernia. There weren’t any overlying skin changes, however, there was tenderness on palpation. His vital signs were stable, initial haematological and biochemical workup was done in the emergency department which included a full blood count, urea, creatinine and electrolytes along with C- reactive protein levels; all these tests were unremarkable.

The patient was prepared for open surgery, with the intention of doing a routine right inguinal hernia repair with an onlay mesh keeping with the past history without any major co-morbidities. Pre-operatively, the patient was given antibiotics for surgical prophylaxis.

Under general anaesthesia, the right inguinal canal was opened and the cord was delivered along with the sac and its contents. Upon opening the hernia sac, a large indirect hernial sac containing a long loop of sigmoid colon with an inflamed epiploica was seen. This is seen in Figure 1, as the sac is opened and the contents are displayed showing the sigmoid colon with the tinea running down, the inflamed appendage is seen; Figure 2 and 3 show the inflamed appendage without any gangrenous changes as highlighted by the forceps. As the appendage appeared thickened and inflamed, it wasn't resected but in fact reduced back into the abdominal cavity along with the sigmoid colon. A standard, tension-free Lichtenstein repair was performed with a mesh that was anchored using Prolene 2-0 suture. 

**Figure 1:** Operative findings: Sigmoid colon (S) in the sac along with the inflamed epiploic appendage (EA).

**Figure 2:** Operative findings: The forceps showing the inflamed epiploic appendage with the sac below

**Figure 3:** The forceps identifying the inflamed appendage which was later reduced back in the abdominal cavity along with contents

A 16 F Redivac drain was placed over the external oblique aponeurosis and into the right scrotum to prevent seroma formation. 

Normally antibiotics arent given in the postoperative phase however, in this case, were continued for only three doses. This decision was taken into consideration due to the operative findings (inflamed epiploica) along with the comorbidities the patient had, there was a risk of him developing a wound infection, hence, antibiotics were given for three postoperative doses.

The drain was removed on the second postoperative day after the output had reduced to less than 20 ml/day. The patient did not suffer from any postoperative complications and was discharged on the second postoperative day.

## Discussion

The perioperative findings of an inflamed epiploic appendage of the sigmoid colon within an incarcerated inguinal hernial sac on the right side led us to conduct a web search. We came across five publications of epiploic appendagitis of the sigmoid colon within a groin hernia, all of which were thoroughly reviewed. Other articles identifying epiploic appendages from the references of the articles were reviewed. During the search, we found the association of epiploic appendage in a hernial sac reported by Hunt as early as 1919 [3]. The presentation could either be in the form of strangulation or torsion of the appendage [4]. Demographics were not published for another case. 

Our case matched most of the studies mentioned above with regards to patient demographics, as the majority of cases were in men aged 60 and above [5-8]. The clinical presentation of pain and swelling was common to prior reports as well as our own. The literature review also identified most cases of EA within a hernia involved the sigmoid colon and occurred in left inguinal hernias, this was contrary to our findings of the hernia being on the right side (this may have been due to a long tortuous sigmoid colon). In addition to this, all patients had an uneventful recovery postoperatively including ours.

However, unlike the majority of the other cases, not only did we find the hernia on the right side (it is atypical as one would find the sigmoid colon herniating through the left groin instead of the right side), but also, we did not resect the appendage at the time of surgery as the tissues were oedematous and swollen and the appendage was not gangrenous. Any further dissection down in this area of inflammation would have posed more risk than benefit to our patient, especially with regards to bowel perforation. This risk would have also been compounded by the small diverticula hiding in the appendage. We replaced the hernial contents, repaired the defect and re-enforced the inguinal wall with a flat mesh. As it was a large and long-standing hernia, a redivac drain was placed in the dead space to evacuate any postoperative haematomas or seromas.

Vesalius first described epiploic appendages in 1543 as anatomic entities along the antimesenteric border of three ribbon-like structures called taenia coli. Tinea libera, mesocolica and omentalis are located anteriorly, posteromedial and posterolateral respectively, running their way from the caecum to the sigmoid colon. The adult colon has 50 to 100 epiploic appendages, which are small serosa-covered, fat-filled outpouchings present on the external surface of the colon. Although these appendages can occur throughout the large bowel, they are most commonly located in the sigmoid colon. This is likely why over 50% of cases of EA involve the sigmoid colon [9]. The appendages are hypothesised to have a protective effect on bowel blood supply during peristalsis and contribute to immunity. They contain branches of arteries, veins and lymph nodes that supply and drain the respective colonic region. EA occurs when these outpouchings become inflamed. The primary form of this condition occurs due to ischemic infarction of the appendage, caused by torsion or spontaneous thrombosis of the epiploic appendage central draining vein [9]. EA has been identified in 2-7% of patients suspected to have diverticulitis and 0.3-1% of those suspected to have appendicitis. In such a presentation, the appendages may become inflamed by being in the vicinity of an ongoing inflammatory process, causing the secondary form of this condition [10]. EA is rare, with an estimated incidence of only 8.8 per million patients per year and a frequency of occurrence of 1.3% [11]. However, we may not know the exact incidence of EA and suspect it may be underreported. Furthermore, as diagnostics are improving, we have a greater inclination towards performing diagnostic laparoscopy for non-specific abdominal pain, increasing our likelihood of detecting this condition [6]. At present, CT scans are the best way of diagnosing EA. Key findings include stranding around the appendage and mesentery, hyperdensity and thickening of the parietal peritoneum [10]. A suspected diagnosis of acute appendicitis, acute diverticulitis, or omental infarction would be the list of differentials that need to be ruled out without an obvious hernia in cases of patients presenting with lower abdominal pain and tenderness. In most cases, non-contrast CT can help distinguish between these entities. Primary EA usually does not require surgical intervention and self-resolves in two weeks with conservative management, such as the use of non-steroidal anti-inflammatory drugs [6]. Therefore, mistaking EA for an acute surgical diagnosis may lead to unnecessary surgery. Greater awareness regarding this condition and CT as a mode of diagnosis is required amongst clinicians. However, it is also important to note that CT cannot always confidently distinguish EA from other surgical pathologies such as diverticulitis. This was seen in the case reported by Özkurt et al. [6]. Our patient required emergency surgery as his hernia became irreducible, with EA being discovered as an incidental finding. Doing a CT scan would have been inappropriate as it would have delayed the required surgical intervention.

## Conclusions

An irreducible incarcerated inguinal hernia warrants an emergency operation. However, it would naturally take the surgeon by surprise to discover epiploica in an incarcerated hernial sac. This incidental finding has the potential to complicate matters further with regard to management. As it is not routine to scan all patients with this presentation, it is nearly impossible to be aware of this rare picture preoperatively. In addition, prior knowledge of EA in an incarcerated hernial sac would not dissolve the need for an emergency operation. However, this case highlights the importance for the surgeon to remain open-minded regarding the site of the hernia and contents of the sac whether it is an appendix, Meckel's diverticulum or colon with EA. In all these scenarios, the outcome of potential resection and repair would remain the same. In our case, the inflamed appendage was not gangrenous, it was hence returned back to the abdominal cavity and the hernia was repaired through standard technique. This just highlights another approach in the management of EA that differs from resection.
